This article has been retracted.

# The Role of Scleraxis in Fate Determination of Mesenchymal Stem Cells for Tenocyte Differentiation

**DOI:** 10.1038/srep13149

**Published:** 2015-08-20

**Authors:** Yonghui Li, Melissa Ramcharan, Zuping Zhou, Daniel J. Leong, Takintope Akinbiyi, Robert J. Majeska, Hui B. Sun

**Affiliations:** 1 Leni and Peter W. May Department of Orthopedics, Mount Sinai School of Medicine, New York, NY 10029; 2 Department of Biomedical Engineering, City College of New York, New York, NY 10031; 3 Department of Orthopedic Surgery, Albert Einstein College of Medicine, Bronx, NY 10461; 4 Department of Radiation Oncology, Albert Einstein College of Medicine, Bronx, NY 10461.

## Abstract

Mesenchymal stem cells (MSCs) are pluripotent cells that primarily differentiate into osteocytes, chondrocytes, and adipocytes. Recent studies indicate that MSCs can also be induced to generate tenocyte-like cells; moreover, MSCs have been suggested to have great therapeutic potential for tendon pathologies. Yet the precise molecular cascades governing tenogenic differentiation of MSCs remain unclear. We demonstrate scleraxis, a transcription factor critically involved in embryonic tendon development and formation, plays a pivotal role in the fate determination of MSC towards tenocyte differentiation. Using murine C3H10T1/2 pluripotent stem cells as a model system, we show scleraxis is extensively expressed in the early phase of bone morphogenetic protein (BMP)-12-triggered tenocytic differentiation. Once induced, scleraxis directly transactivates tendon lineage-related genes such as tenomodulin and suppresses osteogenic, chondrogenic, and adipogenic capabilities, thus committing C3H10T1/2 cells to differentiate into the specific tenocyte-like lineage, while eliminating plasticity for other lineages. We also reveal that mechanical loading-mediated tenocytic differentiation follows a similar pathway and that BMP-12 and cyclic uniaxial strain act in an additive fashion to augment the maximal response by activating signal transducer Smad8. These results provide critical insights into the determination of multipotent stem cells to the tenocyte lineage induced by both chemical and physical signals.

Mesenchymal stem cells (MSCs) can give rise to mesenchymal lineages such as osteocytes, chondrocytes, and adipocytes, and potentially transdifferentiate into non-mesenchymal cell types such as pancreatic cells and cardiomyocytes^1^,^2^,^3^,^4^. MSCs are considered the ideal source of cellular therapeutic agents for tendon repair^5^,^6^,^7^,^8^. Although increasing studies show that MSCs can be induced to differentiate into tenocytes^5^,^9^,^10^, the potential regulators that govern MSC fate for tenocyte differentiation in tendon neoformation and regeneration have not yet been defined. A number of growth factors, particularly members of the bone morphogenetic proteins (BMP) family, have been shown to promote tenocytic differentiation from the multipotent MSCs^9^,^11^,^12^. Of the more than 20 BMP members^13^, BMP-12 appears to be the most potent tendon inducers identified thus far. BMP-12 gene transfer augments the repair of lacerated tendon^9^,^14^ and improves Achilles tendon healing^15^. *In vitro*, bone marrow MSCs transfected or stimulated with BMP-12 exhibit efficient generation of tenocyte-like cells^6^,^16^. In addition to chemical factors, stimulatory effects of mechanical loading on the tenocytic differentiation have also been described^17^,^18^,^19^. Despite these efforts, however, the molecular mechanisms responsible for the directed differentiation of MSCs into tenocytes are not well understood.

During embryogenesis, many transcriptional factors such as Six1 and Six2, EphA4, Eya1 and Eya2, follistatin, tenascin, mohawk, and scleraxis are recognized to regulate tendon development and formation^20^,^21^,^22^. Among them, scleraxis a class II basic helix-loop-helix (bHLH) transcription factor, has received particular attention^23^. Scleraxis (Scx) is expressed in both stem cells and differentiated cells of tendons. At E10.5 endogenous Scx can be readily detected in the developing limb buds and in a somatic compartment known as syndetome at the dorsolateral edge of the sclerotome^24^,^25^,^26^, and its expression is continued throughout later stages of tendon formation^24^. Conditional knockout of the *Scx* gene in mice causes a failure in the condensation of tendon stem cells and severe defects in tendon differentiation, and consequently a dramatic loss of tendons that are particularly responsible for transmitting musculoskeletal force in the limbs, tail and trunk^27^. These studies highlight an essential role of Scx in tendon development, and suggest that Scx may be critically involved in fate determination of adult MSCs to differentiate into tenocytes.

Here we showed that Scx is a key regulator of MSC differentiation into the tenocyte lineage as evidenced by its critical involvement both in the activation of downstream genes and suppression of non-tenogenic pathways in C3H10T1/2 cells. Our study provides evidence suggesting that the tenocytic differentiation process of adult MSCs may recapture the molecular cascades operative in embryonic tendon formation.

## Results

### Scleraxis is induced by BMP-12 in C3H10T1/2 cells

To investigate the involvement of Scx in the tenogenic differentiation of MSCs, we first determined whether BMP-12 would induce Scx in C3H10T1/2 stem cells. As assessed by RT-qPCR, BMP-12 treatment led to strong expression of *Scx* and Tenomodulin (*Tnmd*), a marker related to later stage tendon formation^28^. The induction of both genes were dependent on the dose of BMP-12; increases in expression of *Scx* and *Tnmd* were detectable at 2.5 ng/ml and maximal (2.5 ~ 3-fold over untreated controls) at 10–25 ng/ml (Fig. 1A). Simultaneously, BMP-12 downregulated the expression of neucleosteimin (*Nst*), a pan-stem cell marker (Fig. 1B). Tnmd is subject to positive regulation by Scx in a tendon cell lineage-dependent manner^28^. Consistent with this behavior, induction of *Tnmd* lagged behind induction of *Scx* following BMP-12 treatment, as evidenced at the mRNA level by RT-qPCR (Fig. 1C) and at the protein level by immunostaining (Fig. 1D).

### Scleraxis is required for tenomodulin expression in C3H10T1/2 cells

Based on the sequential expression of *Scx* and *Tnmd* pattern and previous findings that Scx stimulates Tnmd expression^28^, we next determined whether *Tnmd* expression in C3H10T1/2 cells could be directly regulated by *Scx* by examining *Tnmd* expression under conditions of *Scx* gain- and loss-of-function. In transient transfection assays, C3H10T1/2 cells overexpressing *Scx* showed significantly upregulated *Tnmd* compared to untransfected and empty vector-transfected cells (Fig. 2A), providing evidence that simply increasing the level of Scx can mimic the inductive effect of BMP-12. On the other hand, when *Scx* expression was suppressed by transfection with *Scx* siRNA, the BMP-12-dependent upregulation of both *Scx* and *Tnmd* seen in untransfected and scrambled siRNA-transfected cells was abolished (Fig. 2B). Furthermore, while transfection with *Tnmd* siRNA blocked BMP-12-induced *Tnmd* expression, it had no effect on expression of *Scx* (Fig. 2B). Similar results were also obtained at protein levels by Western blotting (Fig. 2C).

### Scleraxis directly transactivates tenomodulin in C3H10T1/2 cells

Scx modulates the expression of target genes by binding to a consensus sequence (CANNTG) called E-box within promoters^29^. To test whether Scx might directly transactivate the transcription of Tnmd via this mechanism, we carried out electrophoretic mobility shift assays (EMSA) using olgionucleotide probes containing a putative E-box and sequences from the Tnmd promoter flanking both sides of the E-box. As shown in Fig. 3A, a protein-DNA complex was detected only when probes were incubated with nuclear extracts prepared from cells expressing high levels of Scx due to transfection (Fig. 3A, lane 3) or BMP-12-treatment (Fig. 3A, lane 4). The shifted bands became undetectable in the presence of excess unlabeled wild-type (Fig. 3A, lane 6, 7) or mutant probes (Fig. 3A, lane 9, 10). To identify specific E-box sites in the Tnmd promoter that interact with Scx, we further conducted chromatin immunoprecipitation (ChIP) assays. Of the five putative E-boxes found within the −3000 bp region of the Tnmd promoter, E-boxes 1 to 4, but not E-box 5, demonstrated functional interactions with Scx (Fig. 3B).

### Scleraxis promotes tenocytic differentiation by suppressing non-tenogenic potentials of C3H10T1/2 cells

Loss of *Nst* expression in C3H10T1/2 cells stimulated by BMP-12 suggests that tenocyte differentiation may be associated with loss of stem cell features, which are likely reflected by a decline in the capacity to differentiate along alternative pathways. Therefore, we next determined whether Scx was involved in the suppression of non-tenogenic potential. RT-qPCR analysis showed in C3H10T1/2 cells plated at colony-forming densities and treated with varying concentrations of BMP-12, *Scx*-expressing colonies increased in a BMP-12 dose-dependent manner (Supplementary Fig. S1), although not all of them expressed *Scx*.

We further tested whether Scx-positive (Scx^+^) and Scx-negative (Scx^−^) colonies differ in their differentiation potentials using a single CFU-F re-plating assay (SCRA) (Fig. 4A). When cells from individual Scx-positive (Scx^+^) and Scx-negative (Scx^−^) colonies were re-plated in lineage-specific induction media, cytochemical staining for lineage specific markers revealed that the osteogenic, chondrogenic and adipogenic differentiation were largely suppressed in Scx^+^ colony-derived cells, but maintained in cells from Scx^−^ colonies (Fig. 4B,C). These results were further confirmed by assessing mRNA levels of lineage-specific genes (Fig. 4D).

To test a direct role for Scx and/or Tnmd in suppressing non-tenocytic activities, the loss of function of both genes were examined. As shown in Fig. 5, marked increases in the expression of osteo-, chondro-, and adipose-specific genes were detected in *Scx* siRNA transfected cells in the presence of induction media. The expression of these genes was increased in untransfected and scrambled siRNA transfected cells that received BMP-12 treatment to induce *Scx* prior to lineage induction, or in those without induction. These data show Scx is a negative regulator of the osteogenic, chondrogenic, and adipogenic pathways. Notably, silencing of *Tnmd* in the presence of high levels of *Scx* did not fully suppress non-tenogenic gene expression, especially chondrocyte- and adipocyte markers, showing that Tnmd may also participate in suppression of non-tenocytic potentials.

### Combining cyclic loading and BMP-12 enhances expression of Scx and formation of tenocyte-like cells

Mechanical stress has been shown to influence tenocytic differentiation from MSCs *in vitro*^19^,^30^ and from tendon stem and progenitor cells *in vivo*^18^,^31^,^32^,^33^,^34^. Therefore, we further tested whether mechanical loading also modulates tenocyte differentiation in C3H10T1/2, and whether such a physical stimulus can act synergistically or additively with BMP-12. We first assessed the effects of cyclic uniaxial strain loading on *Scx* expression. Compared to non-loaded controls, significant increases in *Scx* expression were observed in all loading-stimulated groups of cells with maximal expression in cells loaded at 5% strain (Supplementary Fig. S2A) at 0.5 Hz (Supplementary Fig. S2B).

We next examined the combined effects of BMP-12 and stretch loading. Consistent with experiments described above, both mechanical loading and BMP-12 treatment resulted in significant increases in *Scx* mRNA expression though the latter provoked a more pronounced response. When the two stimuli were applied simultaneously, however, the increases in gene expression appeared to be additive (Fig. 6A). Toluidine blue staining revealed that cells treated with a combination of mechanical loading plus BMP-12- appeared to resemble more closely mature tenocytes (Fig. 6B) as evidenced by a greater elongation (Fig. 6C) and cell alignment (Fig. 6D). The data show that physical and biochemical signals can interact cooperatively to facilitate differentiation into tenocytic cells.

### Smad8 is an upstream signaling molecule of Scx required to mediate the teno-inductive response of cyclic loading and BMP-12

Members of the receptor-regulated Smads (R-Smads) subclass, Smad1/5/8, are the major signaling transducers for BMPs^35^. We monitored the phosphorylation of these proteins in cells under different treatment conditions. While BMP-12 and stretch loading each induced extensive phosphorylation of Smad 1/5/8, significantly increased R-Smad phosphorylation was observed over the two time-points in cells that had received both stimuli (Fig. 7A). The data demonstrate that BMP-12 and mechanical loading signaling may interact at the R-Smad site, thus leading to augmentation of tenocytic differentiation.

To pinpoint the Smad molecule specifically involved in the mechanical loading and BMP-12 induction of *Scx*, we assessed the effects of Smad1, Smad5 or Smad8 suppression. Phosphorylation of Smad 1/5/8 mediated by BMP-12, loading, or both, was almost entirely repressed upon Smad8 knockdown by siRNAs (Fig. 7B), concurrent with absence of *Scx* induction associated with the treatments (Fig. 7C). In contrast, Smad1 or Smad5 knockdown (Fig. 7D) had minimal impact on the overall phosphorylation of Smad 1/5/8 (Fig. 7E).

## Discussion

Stem cell-based approaches are considered to have a great potential to improve healing of soft tissue injuries, which account for nearly half of the 33 million musculoskeletal injuries that occur in the United States each year^36^. The effective use of MSCs relies on a better understanding of the signaling pathways that control their differentiation into tenocytes. In the present study, we have demonstrated for the first time that scleraxis, a class B bHLH transcription factor, is critical in determining the fate of C3H10T1/2 stem cells to commit to a tenocyte lineage.

We showed that the induction of Scx was a key early event occurring in the BMP-12-mediated tenocytic differentiation of C3H10T1/2 cells and required to regulate the expression of downstream gene Tnmd, a well characterized marker related to a late stage of tenocyte differentiation^28^. This conclusion was supported by several lines of evidence. First, treatment with recombinant BMP-12 proteins led to sequential expression of *Scx* and *Tnmd* in C3H10T1/2 stem cells. Second, overexpression of *Scx* in C3H10T1/2 cells simulated the effect of BMP-12 on the upregulation of *Tnmd* whereas knockdown of *Scx* abolished BMP-12 induced *Tnmd*, indicating that the advent and presence of *Scx* is substantive to the ensuing expression of *Tnmd*. Third, altering the expression levels of *Tnmd* had minimal impact on *Scx* induction as demonstrated in comparable experiments on *Tnmd* gain- and loss-of-function. Finally, Scx directly transactivated Tnmd, a process entailing the recruitment and binding of Scx to the multiple selective E-boxes within the promoter region of Tnmd. Although we have not examined other later markers along the teno-differentiation such as type I collagen genes and aggrecan, Scx may also be poised to modulate the expression of these genes as well^29^,^37^,^38^. Our previous study demonstrated that BMP-12 treatment of rat adult MSCs derived from bone marrow (BM-MSCs) induces these adult stem cells undergoing tenocyte differentiation, as remarked by expression of not only *Scx* and *Tnmd*, but also other late teno-phenotypic markers collagen I and tenascin C^9^. The BMP-12 treated MSCs showed ability in augmenting tendon-like tissue formation and defect repair *in vivo*. Together, these studies suggest induction of Scx is a key early event in BMP-12-mediated tenocyte differentiation in both embryonic-derived (i.e. C3H10T1/2) and adult (i.e. BM-MSCs) MSCs.

In addition to its indispensable role in the control of downstream genes within the tenogenic pathway, Scx might also be directly responsible for the suppression of non-tenocytic differentiation potentials of C3H10T1/2 cells. Utilizing a sophisticated approach combining single colony-forming assay and RT-qPCR, we were first able to identify and successfully separate two types of colonies: Scx^+^ and Scx^-^ colonies, and found that while the osteogenic, adipogenic, and chondrogenic capabilities were largely abrogated in Scx-positive cells, all of those distinct lineage potentials were, surprisingly, well maintained in Scx-negative cells. The inhibitory role of Scx was collaborated by the observation that upon repression of Scx by siRNA, C3H10T1/2 cells were capable of retaining their multi-lineage potentials even in the presence of BMP-12, which was exactly the same as those observed with Scx^-^ cells. In support of our data, reports documented that Scx and Sox9, a master transcription factor for chondrogenesis^39^,^40^, are co-expressed in sclerotome during the early stage of embryonic development, but Scx is markedly reduced in the center of Sox9-expresssed sclerotome following development^41^, underlining a potentially suppressive function for Scx in the chondrogenesis.

It should be pointed out, however, that Scx alone appeared to be insufficient to drive MSC differentiation into tenocytes. Scx^+^ colony-derived cells still expressed osteo-, chondro-, and adipogenic potentials at low but detectably greater levels than un-induced controls (Fig. 4D). We observed a similar phenomenon in cells where only Tnmd, but not Scx, was silenced with siRNA (Scx^+^ Tnmd^-^ cells) (Fig. 5). Most likely, the Scx^+^ colonies derived from single colony-forming assays may harbor Scx^+^ Tnmd^−^ and Scx^+^ Tnmd^+^ sub-fractions, and the former are responsible for the low level of differentiation along non-tenogenic pathways. Given these considerations, we propose that the phenotypic plasticity of C3H10T1/2 cells becomes progressively limited during tenocytic differentiation, and that these changes occur in stages that are functionally determined by the sequential expression of Scx and Tnmd. In the earlier stage, Scx appears to play a central role both in triggering the expression of tenocyte-associated genes (Tnmd and possibly type I collagen, tenascin-C, type XIV collagen), as well as in suppressing non-tenogenic capacity. At the later (Scx^+^/Tnmd^+^) stage, cells become fully committed to the tenocyte phenotype and completely lose their capacity to differentiate into non-tenocyte lineages, at least under the conditions we examined.

The critical role of Scx in tenocyte differentiation of C3H10T1/2 cells was not limited to induction by BMP-12, but was also required for mechanical load-triggered tenocytic differentiation. Moreover, combination of the biochemical and mechanical stimuli led to marked augmentation of the differentiation response incurred by either stimulus alone as evidenced by increased *Scx* expression and enhanced formation of tenocyte-like cells. Furthermore, we found that both BMP-12 and stretch loading induced extensive phosphorylation of Smad8 but differed in the time course of this biochemical process. The mediation of both BMP-12 and stretch loading responses by the Smad system provides a molecular basis to explain not only the crosstalk between these stimuli in controlling tenocyte differentiation, but also the downregulation of non-tenogenic potency by Scx since Smad8 has been shown to promote neotendon formation by inhibiting the osteogenic pathway induced by BMP-2^42^. Together, this study suggests that Smad8 is a key signaling molecule whose activation is required to mediate Scx expression and ensuing tenocytic differentiation of C3H10T1/2 cells in response to BMP-12 and stretch loading.

In summary, we have identified scleraxis as a central regulator responsible for the fate determination of C3H10T1/2 cells to differentiate into tenocytes and suppress alternate pathways for differentiating into other lineages. Both actions are induced by mechanical as well as chemical stimuli that are mediated intracellularly by phosphorylation of Smad8 and act in an additive fashion. These findings offer novel insights into the molecular cascades underlying tenocyte differentiation from pluripotent stem cells, and may contribute to the development of cell-based tissue engineering approaches useful for tendon repair.

## Methods

### Cell culture and stimulation

Murine pluripotent mesenchymal stem cells C3H10T1/2 (ATCC CCL226)^43^ were grown as monolayers in DMEM with 10% fetal bovine serum. Twenty-four hours prior to BMP-12 treatment or mechanical loading, cells were starved for 12 hours in DMEM supplanted with 1% FBS. For BMP-12 treatment, cells were treated with indicated concentration of recombinant mouse BMP-12 (R&D Systems) or PBS (control) in starving media for an additional 12 hours. For mechanical loading, cells were subjected to uniaxial cyclic loading for 1 hour with indicated load levels using a custom-designed cell-loading device connected to a computer controlled linear stepper motor (Anaheim Automation). For combined treatment experiments, cells were treated with BMP-12 for 11 hours and then further treated with BMP-12 for one more hour or subjected to uniaxial cyclic loading for 1 hour at indicated load levels. Following treatments, cells were maintained for an additional 3 to 7 days and collected for analysis of gene expression and morphological changes.

### Single CFU-F replating assay (SCRA)

To determine the differentiation potential of Scx^+^ and Scx^−^ cells derived BMP-12 treated stem cells, SCRA was performed as previously described (20). Briefly, cells were seeded at low density (1 × 10^3^/100 mm culture dish) and cultured for two weeks. Individual colonies were collected with EDTA–trypsin. Cell suspensions from each colony were divided into four portions: one of them was used to assay *Scx* expression by RT-qPCR, and the remaining three portions of cells were replated in individual wells of a 48-well plate containing either osteogenic, chondrogenic, or adipogenic differentiation medium. The osteogenic induction cocktail consisted of growth media supplemented with 10 nM dexamethasone, 50 μg/ml ascorbate-phosphate, and 10 mM β-glycerophosphate (Sigma). The adipogenic induction cocktail consisted of growth media supplemented with 0.5 uM hydrocortisone, 100 μg/ml isobytulmethylxanthine, and 60 μM indomethacin (Sigma). For chondrogenic induction, cells were grown in a micromass culture. 1 × 10^6^ cells were centrifuged in a polypropylene tube at 150 g for 5 min to form a cell pellet. The pellet was suspended in a chondrogenic induction cocktail consisting of growth media supplemented with 10 ng/ml TGF-β3, 50 mg/ml insulin-transferrin-selenium (ITS) + Premix (Invitrogen), and 50 ug/mL ascorbate-phosphate. Cells were harvested after two weeks lineage induction and assayed for osteo-, chondro-, or adipo-phenotype markers gene expression using RT-qPCR or in some cases by immunocytochemical staining.

### Immunocytochemical staining (ICC)

Cells were fixed in 10% formaldehyde, treated with serum-free protein blocking solution (Dako), and then incubated overnight at 4 °C with antibodies against Scx (1:150, Abcam, Rabbit polyclonal), Tnmd (1:150, Santa Cruz Biotechnology, Goat Polyclonal), Runx2 (1:200, Abcam, Rabbit polyclonal), Sox9 (1:200 Santa Cruz Biotechnology, Rabbit polyclonal), PPARγ2 (1:200, Abcam, Rabbit polyclonal), or aggrecan (1:200, Abcam, Rabbit polyclonal). Cells were then rinsed in PBS. For Scx and Tnmd staining, cells were incubated with anti-rabbit Alexafluor 488 (1:1000, Invitrogen) or anti-goat Alexafluor 568 (1:1000, Invitrogen). For the other antibodies, cells were incubated for 30 minutes with anti-rabbit secondary antibody conjugated with horseradish peroxidase (Dako) followed by DAB chromagen (Vector Laboratories) for 2 minutes. Negative control sections were prepared using irrelevant isotype matched primary antibodies (Dako).

### Cytochemical Staining (CCS)

Osteogenic, adipogenic and chondrogenic differentiation were assessed by staining with Alizarian Red S (Sigma) for calcium deposition, Oil Red O (Sigma) and Safranin-O, respectively^44^. Imaging was performed using a Zeiss inverted microscope, Axiocam camera and Axiovision 4.6 software.

### Electrophoretic mobility shift assay (EMSA)

Nuclear extracts of C3H10T1/2 cells—either transfected to overexpress *Scx*, treated with 10 ng/ml BMP-12 or left untreated—were incubated with olgionucleotide probes containing a specific E-box consensus sequence. Probe sequences were 18 bp long and contained the 6-mer E-box consensus sequence (CANNTG) flanked by 6-mer sequences on each side of the E-box to increase the probe’s specificity. Probes were labeled with [α-^32^P] dCTP (PerkinElmer Life Sciences) for detection. Specific binding was assessed by competition with an excess of the unlabeled, wild-type (CANNTG) probes and mutated (CANNTG→AATTTA) probes.

### Chromatin immunoprecipitation (ChIP) assay

C3H10T1/2 cells were treated with 10 ng/ml BMP-12 to induce *Scx* expression or left untreated (control). The ChIP assay was performed using a commercial kit (USB Corporation) following the manufacturer’s instructions. Briefly, cells were treated with 1% formaldehyde to cross-link the scleraxis molecules bound to DNA, and cells were then lysed and sonicated. The samples were immuno-purified using Scx antibodies (Abcam). The subsequent samples were then heated to reverse DNA-protein cross-links and DNA was recovered by phenol/chloroform extraction and resuspended in 10 mM Tris-HCl buffer. Purified DNA was PCR amplified using primer sets designed to include individual E-box sequences with the following priemrs: E-box1 (from start codon): F, 5-CTGAGTTTGCGATTTCTGAGTT-3; R, 5-CTCGATTCTGTGCCTGTAACC-3. E-box2: F, 5-AAGAAAGCAAGCTGGAGGAA-3; R, 5-GAGCATCTGTACCCGGATGT-3. E-box3: F, 5-CGTTTCTTCTTCCTTCCTTCC-3; R, 5-ACCTCACCCTTCCCTGTCTT-3. E-box4: F 5-TGTATATTATGGTTTCCAATG-3; R, 5-GAAGGAAGGAAGAAGAAACG-3. E-box5: F, 5-TGTGTTTCTCCAGGGGAGTC-3; R, 5-CACACACACACTGTGCCAAA-3.

Total RNA isolation, Reverse transcription and quantitative PCR (RT-qPCR).  Total RNA was isolated using the RNeasy Mini Kit (Qiagen). Reverse transcription was carried out using oligodT and Superscript II (Invitrogen). RT-qPCR was performed with a SYBR Green PCR Master Mix (Applied Biosystems) using ABI Prism 7900HT sequence detection system (Applied Biosystems), and normalized with GAPDH and β-actin levels. The housekeeping genes have been confirmed to be not regulated by stimuli such as BMP-12. Data were analyzed using the threshold cycle (Ct)-relative quantification method. Primer pairs used in this study are listed in Supplementary Table S1.

### Overexpression of Scx and Tnmd

Enforced expression of *Scx* and *Tnmd* were performed by transfecting C3H10T1/2 cells with vectors containing the coding region of murine *Scx* or *Tnmd*, or with no insert using Lipofectamine 2000 reagent (Invitrogen). Cells were then analyzed for *Scx* and *Tnmd* mRNA expression by RT-qPCR.

### siRNA Transfections

siRNA transfections were carried out using Lipofectamine 2000 reagent (Invitrogen) according to the manufacturer’s instructions. C3H10T1/2 cells were transfected with either *Scx*-siRNA, *Tnmd*-siRNA, *Smad1*-siRNA, *Smad5*-siRNA, or *Smad8*-siRNA (Santa Cruz Biotechnologies, Inc., Santa Cruz, CA). Cells were then treated with 10 ng/ml BMP-12 for 12 hours prior to harvest for RT-qPCR or Western blot.

### Western Blot

Cell lysates were prepared using RIPA lysis buffer (Pierce Technologies) and protease and phosphatase inhibitor (Thermo Scientific). Proteins were separated in 12% SDS-PAGE gel and transferred onto a nitrocellulose membrane and blocked with milk protein. Membranes were incubated with anti-Scx (1:1000, Rabbit polyclonal, Santa Cruz Biotechnology), anti-Tnmd (1:1000, Rabbit polyclonal, Santa Cruz Biotechnology), anti-phospho-Smad 1/5/8 (1:1000, Rabbit polyclonal, Millipore), anti-Smad8 (1:1000, Rabbit polyclonal, Santa Cruz Biotechnology), or α-Tubulin (1:1000, Rabbit polyclonal, Santa Cruz Biotechnology) followed by incubation with anti-rabbit conjugated with horseradish peroxidase (Santa Cruz Technologies). Membranes were washed with TBST and immunoreactivity was normalized by chemiluminescence using ECL Plus Detection system (Amersham Biosciences).

### Statistical analysis

The data were expressed as mean ± S.D. Statistical comparisons between two groups were performed using Student’s *t*-test or one-way ANOVA with Tukey post-hoc test (for RT-qPCR results)*. p* < 0.05 was considered statistically significant.

## Additional Information

**How to cite this article**: Li, Y. *et al*. The Role of Scleraxis in Fate Determination of Mesenchymal Stem Cells for Tenocyte Differentiation. *Sci. Rep*. **5**, 13149; doi: 10.1038/srep13149 (2015).

## Supplementary Material

Supplementary Information

## Figures and Tables

**Figure 1:** Induction of scleraxis and tenomodulin by BMP-12 in C3H10T1/2 stem cells. (**A**) Upregulation of *Scx* and *Tnmd*. (**B**) Downregulation of *Nst* Expression. Cells were left untreated or treated with different concentrations of BMP-12 for 24 hours. mRNA levels were determined by RT-qPCR. Data are expressed as mean ± S.D. (*n* = 6). *p < 0.05. (**C**,**D**) Time course of *Scx* and *Tnmd* expression. Cells were treated with 10 ng/ml of BMP-12 for different lengths of time. mRNA (**C**) and protein (**D**) levels of gene expression were determined by RT-qPCR and immunostaining, respectively. Data in (C) are expressed as mean ± S.D. (*n* = 3).

**Figure 2:** Scleraxis-dependent expression of tenomodulin in C3H10T1/2 cells. (**A**) Overexpression of *Scx* upregulated *Tnmd*. Cells were left untransfected or transiently transfected with empty vectors or vectors containing *Scx* or *Tnmd* cDNA. mRNA levels were determined by RT-qPCR. Data are expressed as mean ± S.D. (*n* = 3). *p < 0.01. (**B**,**C**) Knockdown of *Scx* blocked BMP-12-induced *Tnmd*. C3H10T1/2 cells untransfected or transfected with scramble siRNA, or *Scx* siRNA, or *Tnmd* siRNA were left untreated or stimulated with BMP-12, and mRNA and protein levels of gene expression were determined by RT-qPCR and Western blot, respectively. Data in (**B**) are expressed as mean ± S.D. (*n* = 6). *p < 0.05.

**Figure 3:** Transactivation of tenomodulin by scleraxis in C3H10T1/2 cells. (**A**) Binding of Scx to Tnmd E-boxes assessed by electrophoretic mobility shift assays (EMSA) Olgionucleotide probes corresponding to a specific E-box consensus sequence were incubated with nuclear extracts from C3H10T1/2 cells with either *Scx* overexpression and/or BMP-12 treatment or left untreated (control). (**B**) Binding of Scx to Tnmd E-boxes assessed by chromatin immunoprecipitation (ChIP) assays. Cross-linked chromatins were prepared by immuneprecipitated cellular lysates using anti-scleraxis antibodies and purified DNA was used to PCR amplify the biding regions of *Tnmd* promoter. The binding of Scx to all tested *Tnmd* E-boxes except 5 was detected in BMP-12-treated cells. Upper panel, distribution and localization of E-boxes in *Tnmd* promoter.

**Figure 4:** Scleraxis induction is associated with loss of non-tenogenic potential of C3H10T1/2 cells. (**A**) Schematic procedures of single CFU-F replating assay (SCRA). (**B**) Cytochemical staining of osteo-(left panel), chondro-(middle panel), and adipo-(right panel) differentiation. (**C**) Immunohistochemical staining of lineage-specific markers. Data shown in B and C are representatives of three experiments. (**D**) mRNA expression of lineage-specific marker genes determined by RT-qPCR. Data are expressed as mean ± S.D. (*n* = 6). *p < 0.01.

**Figure 5:** Scleraxis knockdown preserves multi-potent potentials in C3H10T1/2 cells. Untransfected C3H10T1/2 cells or cells transfected with scramble siRNA, or *Scx* siRNA, or *Tnmd* siRNA were left untreated or treated with BMP-12 for 24 hours and further incubated for designed length of time in the absence or presence of lineage induction media. The phenotypes (*Scx* and *Tnmd* expression) of respective groups of cells and mRNA expression of lineage-specific marker genes were assayed by RT-qPCR. Data are expressed as mean ± S.D. (*n* = 6). *p < 0.05.

**Figure 6:** Compound effects of BMP-12 and cyclic loading on the tenocytic differentiation of C3H10T1/2 stem cells. (**A**) Induced expression of *Scx* by BMP-12 and cyclic stretch loading. Cells were left untreated or treated with BMP-12 alone, or cyclic loading alone, or BMP-12 plus cyclic loading. After incubation, cells were harvested and analyzed for *Scx* mRNA expression by RT-qPCR. Data are expressed as mean ± S.D. (*n* = 3). *p < 0.05. (**B**) BMP-12 and stretch loading induced cell morphological changes. Cells were treated as in (**A**) and stained with toluidine blue. (**C**) Nuclear aspect ratio: width vs length of nucleus; (**D**) Nuclear orientation angle: deviation of nuclear axis from average axis. *p < 0.05. *C: Control, B: BMP-12 only, S: stretch loading only, B* *+* *S: BMP-12+stretch loading*.

**Figure 7:** Dependency of Smad8 activation in BMP-12 and cyclic stretch loading signals. (**A**) Enhanced Smad 1/5/8 phosphorylation induced by combined treatment of BMP-12 and cyclic stretch loading. Cells under indicated treatment were harvested at 1 hour and 2 hours post-treatment to analyze the levels of Smad1/5/8 phosphorylation by Western blot. (**B–E**) Activation of Smad8 in C3H10T1/2 stem cells in response to BMP-12 and stretch loading. Cells were transfected with siRNA against *Smad1*, *Smad5*, *Smad8*, or control siRNA, (siScr) followed by treatment of BMP-12 or loading or both, and protein phosphorylation analyzed by Western blot. *C: Control, B: BMP-12 only, S: stretch loading only, B* *+* *S: BMP-12+stretch loading, Scr: Scramble of siRNA, siS1: siRNA-Smad1, siS5: siRNA-Smad5, siS8: siRNA-Smad8*.
